# Interleukin-27 ameliorates coxsackievirus-B3-induced viral myocarditis by inhibiting Th17 cells

This article has been retracted.

**DOI:** 10.1186/s12985-015-0418-x

**Published:** 2015-11-14

**Authors:** Hengshan Zhu, Chuang Lou, Ping Liu

**Affiliations:** Department of Cardiovascular Surgery, Xianyang Hospital of Yan’an University, Xianyang, 712000 Shaanxi China; Department of Cardiology, AnKang Hospital of Traditional Chinese Medicine, Ankang, 725000 Shaanxi China; Department of Cardiology, Xianyang Hospital of Yan’an University, No 38 Wenlin Raod, Xianyang, 712000 Shaanxi China

**Keywords:** Interleukin-27, Viral myocarditis, CVB3, Th17 cells

## Abstract

**Background:**

Interleukin (IL)-27, which has both pro and anti- inflammatory properties, is a new discovered heterodimeric cytokine that belongs to IL-12 family. However, the expression pattern and functional role of IL-27 in viral myocarditis (VMC) has not been investigated.

**Methods:**

BALB/c mice were intraperitoneally (i.p) infected with Coxsackie virus B3 (CVB3) for establishing VMC models. Mice were then injected i.p. with Anti-Mouse IL-27 p28Ab or recombinant IL-27 for neutralization and overexpression of IL-27. The survival rates of mice were recorded and the kinetics of IL-27 expression, the frequencies of Th17 cells and the expression of inflammatory cytokine in CVB3-infected mice were determined by ELISA, real-time PCR and flow cytometry.

**Results:**

The IL-27 expression in heart tissues and serum in coxsackievirus B3 (CVB3)-induced myocarditis mice peaked on day 4 but then rapidly decreased during the late infectious stage of CVB3, high IL-27 levels were negatively correlated with bodyweight loss (*r* = −0.71, *P* = 0.021) and myocardial pathological score (*r* = −0.85, *P* = 0.0018). Additionally, neutralization of IL-27 with Anti-IL-27 Ab accelerated, whereas systemic administration of recombinant mouse IL-27 ameliorated CVB3-induced myocarditis. The protective role of IL-27 in VMC was reflected by an improved survival rate, increased bodyweights, and reduced pathological scores in Anti-IL-27 group compared with IgG control group. Mechanistic investigations showed that IL-27 inhibited Th17 cells frequencies and IL-17 production, as well as the Th17-related proinflammatory cytokines in heart tissues.

**Conclusions:**

Our results demonstrate that that IL-27 effectively protects the myocardium from the pathogenesis of CVB3 induced myocarditis, which may be attributable to reduced Th17 production. IL-27 might serve as a novel therapeutic treatment for VMC.

**Electronic supplementary material:**

The online version of this article (doi:10.1186/s12985-015-0418-x) contains supplementary material, which is available to authorized users.

## Background

Viral myocarditis (VMC), which was characterized by myocardial inflammation and can progress to acute myocarditis, chronic dilated cardiomyopathy and even congestive heart failure, has been recognized as a common cause of abrupt death in young adults [1]. Coxsackie virus B3 (CVB3), an enteric virus of the *Picornaviridae* family, is thought to be the leading cause of VMC [2]. Accumulating evidence had indicated that excessively activated inflammation and autoimmune responses triggered by the viral infection, rather than direct viral infection, are the dominant causes of myocardial cells damage in VMC [3, 4]. Emerging evidences have revealed that several T helper (Th) subsets, such as Th1, Treg and Th17 cells, are involved in the pathogenesis of VMC [5]. However, the fundamental mechanisms responsible for VMC remain largely unknown.

IL-27 is a newly discovered heterodimeric cytokine that belongs to IL-12 family, which is composed of the Epstein-Barr virus-induced gene 3 (EBI3) and the p28 subunit [6]. IL-27 signals through a receptor composed of the common IL-6 receptor chain gp130, used by several other IL-6 and IL-12 family members, and a unique IL-27 receptor α chain (IL-27RA) homologous to the IL-12Rβ2 chain of the IL-12 receptor [7]. IL-27 is produced by dendritic cells, monocytes and endothelial cells. Its receptor has been found on various cell types such as T cell subsets, NK cells, NK T cells, dendritic cells, B cells and mast cells [8]. IL-27 plays a critical role in the early regulation of T helper type 1 initiation, and enhances proliferation of naive CD4^+^T cells and naive B cells [9–11]. It, however, also exerts anti-inflammatory functions by inhibiting the development of Th17 cells and inducing IL-10 producing type 1 regulatory T cells [12–14]. Thus, IL-27 plays both pathogenic and protective roles in given infection and autoimmune disease models.

IL-27 was found recently to be a novel anti-HIV cytokine that inhibits HIV-1 replication in both CD4^+^T cells and macrophages [15, 16]. However, the presence of IL-27 in VMC has not been evaluated. The role of IL-27 in the pathogenesis of VMC is still unclear. In this study, we examined the potential effects of IL-27 on VMC using a murine model of VMC induced by CVB3. The kinetics of IL-27 expression, the frequencies of Th17 cells and the expression of inflammatory cytokine in CVB3-infected mice were determined; neutralizing anti-IL-27 antibodies were used to CVB3-infected mice and the therapeutic effects of this strategy on viral myocarditis were assessed.

## Results

### Expression of IL-27 and IL-27R in VMC

To generate an acute viral myocarditis model, male BALB/c mice were injected i.p. with 10^3^ TCID_50_ of CVB3, as described previously [17, 18]. As expected, the signs of VMC were apparent in CVB3-infected mice, including weakness, coat ruffling, irritability, back arching, lethargy, anorexia and weight loss. The bodyweights of the CVB3-infected mice decreased continuously from day 4 post-infection compared with those of control mice (Fig. 1a). In addition, the myocarditis scores of heart sections showed slight myocardial injury on day 4, but increased obviously in subsequent days (Fig. 1b). In contrast, the myocarditis viral replication (positive strand of CVB3) was detected on day 2; the viral loads (negative-strand of CVB3) peaked on day 4 and rapidly decreased subsequently. On day 7, the viral replication and loads have been dropped to very low levels (Fig. 1c), suggesting that viral infection was not the dominant causes of myocardial cells damage in VMC. We also monitored the animal’s survival after CVB3 infection. 8 of 20 (40 %) mice died in the VMC group. Specifically, on day 6, 7, 8, 10, 11 post infection, there were 1, 1, 2, 2, 2 mice dead in the VMC group. In contrast, none of mice died in the control group (Fig. 1d).

**Fig. 1:** Expression kinetics of IL-27 and IL-27R in VMC. Male BALB/c mice were infected with 10^3^ TCID_50_ of CVB3 at day 0. **a** Body weight was monitored daily until day 10 post-infection. **b** The severity of myocarditis was scored every 2 days until day 10 post-infection using a scale based on foci of mononuclear infiltration and myocardial necrosis. **c** The myocarditis viral replication (positive strand of CVB3) and the viral loads (negative-strand of CVB3) were detected using qRT-PCR. **d** The survival rate of CVB3-infected mice and control mice after CVB3 infection were recorded (*n* = 20 per group). The expression of IL-27 in serum (**e**) and cardiac tissue (**f**) were monitored every two days until day 10 post-infection by ELISA assay. The expression of IL-27R mRNA (**g**) and protein (**h**) levels in cardiac tissue on day 7 post infection. Data are showed as the means ± SEM, Each time point contained three mice. ^***^ *P*<0.001

We then examined the kinetic expression of IL-27 after CVB3 infection. As shown in Fig. 1e and f, plasma IL-27p28 levels and IL-27 protein in cardiac tissues peaked on day 4 but then rapidly decreased during the late infectious stage of CVB3, and the significantly increased level of the IL-27 protein and gene transcripts in the VMC group were observed compared with those in the control group during infectious stage of CVB3 from day 2 (Fig. 1e and f). Additionally, the relative gene and protein expression of IL-27RA, the specific receptor of IL-27, was obviously up-regulated in the VMC group, compared with that in the control group on day 7 post infection (Fig. 1g and h).

### Association between IL-27 expression and disease severity in VMC

To further investigate the role of IL-27 in the pathological processes of VMC, the correlation between IL-27 expression and disease activity, including bodyweight loss and myocardial score were analyzed on day 7 post CVB3 infection. As shown in Fig. 2a and b. The IL-27 gene transcripts level in cardiac tissues was negatively correlated with bodyweight loss (*r* = −0.71, *P* = 0.021) and the myocardial pathological score (*r* = −0.85, *P* = 0.0018). Similar results were observed for the serum IL-27 levels (Fig. 2c and d), suggesting that IL-27 may exert a protective effect against CVB3-induced myocarditis.

**Fig. 2:** Association between IL-27 expression and disease severity in VMC. Male BALB/c mice (*n* = 10) were infected with 10^3^ TCID_50_ of CVB3 at day 0. IL-27 expression levels in cardiac tissues were negatively correlated with body weight loss (**a**) and myocarditis pathological score (**b**) on day 7 post-infection. IL-37 expression levels in serum were negatively correlated with body weight loss (**c**) and myocarditis pathological score (**d**) on day 7 post-infection

### Neutralization of IL-27 exacerbated while administration of rmIL-27 alleviated CVB3-induced myocarditis

Next, we examined the protective role of IL-27 against CVB3-induced myocarditis in vivo. As shown in Fig. 3, the results showed that neutralization of IL-27 with Anti-IL-27 Ab accelerated the development of myocarditis and exacerbated the severity, whereas the administration of rmIL-27 ameliorated CVB3-induced myocarditis. Firstly, the survival rate of the Anti-IL-27 group was significantly declined compared with those in IgG control groups (*P* = 0.024), while mice treated with rmIL-27 group exhibited improved survival rate compared with those in PBS control group (*P* = 0.031, Fig. 3a). Additionally, mice treated with Anti-IL-27 underwent marked and continuous bodyweight loss, while mice received rmIL-27 showed slightly bodyweight loss (Fig. 3b). Consistent with these findings, the pathological myocarditis scores of heart sections were higher in mice receiving Anti-IL-27Ab than those IgG control group, and were lower in mice received rmIL-27compared with those in PBS control group (Fig. 3c and d). There were no significant differences between PBS and IgG control groups regarding the survival rates, bodyweight loss and cardiac pathological scores.

**Fig. 3:** Neutralization of IL-27 exacerbated while administration of rmIL-27 alleviated CVB3-induced myocarditis. Male BALB/c mice were infected with 10^3^ TCID_50_ of CVB3 at day 0; mice were injected i.p. with IL-27 p28Ab or rmIL-27 on day 0 and 5 after CVB3 infection. The survival rates (**a**), body weight (**b**) and the severity of myocarditis (**c** and **d**) were monitored. Each group contained ten mice. Results are presented as the mean ± SEM of three independent experiments. ^*^ *P*<0.05, ^**^ *P*<0.01, ^***^ *P*<0.001, compared with PBS group; ^#^ *P*<0.05, ^##^ *P*<0.01, compared with IgG group

### IL-27 ameliorates CVB3-induced myocarditis by inhibiting Th17 cells

Accumulating evidence had indicated that Th17 cells play an important role in the pathogenesis of CVB3-inducedmyocarditis [19, 20]. Moreover, IL-27 had been reported to be a potent inhibitor of Th17 cells [12]. Therefore, we first explored the splenic Th17 frequencies, the characteristic cytokines, and the transcription factor in cardiac tissues on day 7 after CVB3 infection. As shown in Fig. 4a and b, the percentage of Th17 cells in Anti-IL-27 Ab group was higher than those in IgG control group, and reduced two fold by rmIL-27 treatment compared with those in PBS control group. Similar results were observed for the Th17-associated cytokines (IL-17A and IL-22) and the master transcription factor ROR-γt gene expressions in cardiac tissues (Fig. 4c).

**Fig. 4:** IL-27 ameliorates CVB3-induced myocarditis by inhibiting Th17 cells. **a** Representative FACS profile of Th17 cells in the spleen of CVB3 infection mice treated with rmIL-27 or Anti-IL-27 on day 7 post infection. Cells were gated on CD3^+^CD4^+^ T cells. **b** Statistical analysis of the percentage of Th17 cells. **c** Expression of Th17 cells characteristic cytokines, IL-17A, IL-22, and key transcription factor ROR-γt in cardiac tissues on day 7 after CVB3 infection were detected by qRT-PCR. **d** The serum levels of proinflammatory cytokines IL-17A, IFN-γ, IL-6 and TNF-α in CVB3 infection mice were determined by ELISA. Normal, mice not-infected with the virus. Data are showed as the means ± SEM. ^*^ *P*<0.05, ^**^ *P*<0.01, ^***^ *P*<0.001

Activated inflammation triggered by excessive proinflammatory cytokines are the dominant causes of myocardial cells damage in VMC [3]. Thus we further examined the proinflammatory cytokines levels, such as IL-17A, IFN-γ, IL-6, and TNF-α in serum by ELISA. As shown in Fig. 4d, compared with those in IgG control groups, the levels of IL-17A, TNF-α and IL-6 proteins levels were increased dramatically in the Anti-IL-27 Ab group. In addition, significantly lower levels of IL-17A, IL-6, and TNF-α expression were seen in mice treated with rmIL-27. However, the levels of IFN-γ in the Anti-IL-27 Ab group were also higher than those IgG control group, and no significant difference was detected between rmIL-27 treatment group and PBS control group.

## Discussion

IL-27 has both pro- and anti-inflammatory functions. It can activate STAT1 in naive CD4^+^ T cells, stimulate their proliferation and induce Th1 cell differentiation [21]. However, it also suppresses immune responses through inhibition of the development of Th17 cells and induction of IL-10 production by regulatory Tr1 cells in a STAT1- and STAT3-dependent manner [12, 14]. Therefore, its role in VMC, if any, was difficult to predict.

Here we report that IL-27 plays an important role in the pathogenesis of VMC in a CVB3-induced myocarditis mouse model. We initially observed that IL-27 was produced during the infectious stage of CVB3. Its levels in serum and cardiac tissues peaked at day 4 and rapidly dropped during the late infectious stage. In line with the kinetics of IL-27 production, the relative gene and protein expression of IL-27RA, the specific receptor of IL-27, was also obviously up-regulated during the infectious stage of CVB3. However, IL-27 exhibited low expression levels and no alteration in the serum and cardiac tissues in control mice, indicating that IL-27 may not contribute to the initiation of VMC. To our knowledge, this observation provides the first demonstration of an association of increased IL-27 serum and cardiac tissues levels and CVB3-induced myocarditis. Furthermore, it is striking that the severity of VMC negatively correlated with serum and cardiac levels of IL-27, suggesting that IL-27 may exert a protective effect against CVB3-induced myocarditis.

Based on the observation that levels of IL-27 and IL-27 receptor were elevated in VMC, as well as the negative association between IL-27 levels and the severity of VMC, we examined the efficacy of IL-27 in the VMC mouse model, with the use of anti- IL-27 antibody and recombinant mouse IL-27, respectively. Our results proved that neutralization of IL-27 exacerbated the severity of CVB3-induced VMC, which was verified by the lower survive rate, continuous bodyweight loss and higher values of pathological myocarditis scores. On the other hand, administration of rmIL-27 significantly alleviated the severity of CVB3-induced VMC in mice, with reduced cardiac injury and an improved survival rate. Interestingly, rmL-27 did not affect the body weight loss and survival in mice not-infected with the CVB3, suggesting that IL-27 itself have no effect on the immune responses in naïve mouse (Additional file 1: Figure S1). Taken together, our results indicate that IL-27 could be a therapeutic cytokine for the treatment of viral myocarditis as well as other inflammatory diseases.

It is well known that the bias of the T-cell immune response markedly affects the severity of myocarditis. Fierce Th1 immune responses play a critical pathogenetic role in the course of VMC, especially in the subacute stage (days 4–14). However, increasing recent evidences indicate that besides Th1 cells, Th17 cells are also involved in the pathogenesis of VMC. Blockade of IL-17A increases the number of Th1 and CD8^+^T cells and IFN-γ levels, while decreases Treg cells and serum levels of IL-6, IL-10, IL-2, and IL-21, which ameliorates the pathological cardiac changes and reduces viral replication [19, 20, 22]. Interestingly, the induction of distinct Th17 populations contributes to sex based differences in the susceptibility to CVB3-induced myocarditis [18]. In addition, there are several reports demonstrated that IL-27 suppresses Th17 responses. IL-27 suppresses IL-17 production from CD4^+^ T cells stimulated with α-CD3/CD28, IL-6, and TGF-β via mainly STAT1-dependent [13]. IL-27 also suppresses production of IL-22, which is important for Th17 effector function [23, 24]. Thus we speculate that IL-27 may contribute to the alleviation of CVB3-induced myocarditis through modulating Th17 cells responses.

In the present study, we observed a reduction in Th17 cells in the spleens of infected mice after rmIL-27 treatment *in vivo*. Th17-associated cytokines (IL-17A and IL-22) and the master transcription factor ROR-γt gene expressions in cardiac tissues were also noticeably decreased after rmIL-27 treatment. We also observed increased Th1 cells in the spleen after IL-27 treatment (data not shown). Additionally, serum levels of IL-17A, TNF-α and IL-6 were also decreased dramatically post rmIL-27 treatment. Thus, we confirmed that the therapeutic effect of IL-27 on CVB3-induced viral myocarditis is partially attributable to the decline in Th17 cells responses.

## Conclusions

In conclusion, our preliminary data demonstrate for the first time that IL-27 may play a myocardium-protective role through the modulating Th17 cells responses in CVB3-induced viral myocarditis. Therefore IL-27 may serve as a new therapeutic candidate for treatment of VMC. Further studies are required to comprehensively explore the therapeutic potential of IL-27 in human systems.

## Materials and methods

### Mice

Male specific pathogen-free BALB/c mice aged 6–8 week old were purchased from the Laboratory Animal Center of Xi’an Jiaotong University (Shaanxi, P.R. China) and were kept in the pathogen-free facility in the experimental animal center of the Yan’an University (Yan’an, China). All animals received humane care according to the criteria outlined in the “Guide for the Care and Use of Laboratory Animals” prepared by the National Academy of Sciences and published by the National Institutes of Health (NIH publication 86–23 revised 1985). The study protocol was approved by the Ethical Committee of Xianyang Hospital.

### Virus

The CVB3 (Nancy strain) was maintained by passage in HeLa cells. The viral titer was determined using a 50 % tissue culture infectious dose (TCID50) assay on HeLa cell monolayers and calculated by the Reed-Muench method. BALB/c mice were infected with an intraperitoneal (i.p.) injection of 0.1 mL of phosphate-buffered saline (PBS) containing 10^3^ TCID_50_ of the virus for establishing VMC model. Mice administered i.p. with PBS were taken as control.

### IL-27 neutralization and overexpression

For *in vivo* IL-27 neutralization, mice were injected i.p. with Mouse Anti-Mouse IL-27 p28Ab (500 μg per mouse, MM27.7B1, BD Biosciences, San Diego, CA, USA) or control Ab (500 μg per mouse, Mouse IgG2a κ Isotype Control, BD Biosciences, San Diego, CA, USA) on day 0 and 5 after CVB3 infection. For administration of IL-27, mice were injected i.p. with rmIL-27 (1 μg per mouse, BioLegend, San Diego, CA, USA) on day 0 and 5 after CVB3 infection. All surviving animals were sacrificed on day 7 post CVB3 infection. The survival rates were recorded. The hearts, spleens and plasma were collected at indicated time.

### Histopathological analysis and myocarditis scoring

The hearts were collected from the CVB3 infected mice on day 7 and fixed in 10 % formalin, then embedded in paraffin. Sections (5 μm thick) were cut and stained with hematoxylin and eosin (H&E). Histopathological change was observed by using light microscopy (Nikon Eclipse E800 Microscope, Kawasaki, Kanagawa, Japan). Pathological scores were graded by two independent pathologists in a double-blinded manner based on the following semi-quantitative scale: 0 = no inflammation; 1 = one to five distinct mononuclear inflammatory foci, with the involvement of 5 % or less of the cross-sectional area; 2 = more than five distinct mononuclear inflammatory foci, or the involvement of over 5 % but not over 20 % of the cross-sectional area; 3 = diffuse mononuclear inflammation involving over 20 % of the area, without necrosis; and 4 = diffuse inflammation with necrosis.

### Flow cytometry

Splenocytes from CVB3 infected mice on day 7 were isolated and suspended in RPMI 1640 containing 10 % fetal bovine serum, splenic cells were gently dispersed through nylon mesh into a single-cell suspension. Red blood cells were lysed by incubation for 3 min in ACK lysis buffer. The cells were collected and resuspended at a density of 1 × 10^6^ cell/mL. The cells were then stimulated for 4 h with PMA (50 ng/mL) and ionomycin (500 ng/mL) in the presence of brefeldin A (10 μg/mL) at 37 °C, 5 % CO_2_ in a 24-well culture plate (Corning Costar, Corning, NY, USA) in RPMI 1640 medium supplemented with 10 % fetal bovine serum. After 4 h incubation, the cells were harvested and stained with FITC-conjugated anti-mouse CD3 antibody and PE- conjugated anti-mouse CD4 antibody (BD Bioscience, San Diego, CA, USA). After the cells were washed, fixed, and permeabilized according to the manufacturer’s instructions (BD Bioscience, San Diego, CA, USA), cells were stained intracellularly with PE-Cy5.5-conjugated anti-mouse IFN-γ antibody, and APC-conjugated anti-mouse IL-17A antibody (BD Bioscience, San Diego, CA, USA). After incubation at 4 °C for 30 min, the samples were washed in staining buffer and measured on a FACS-Calibur flow cytometer. The data were analyzed using FlowJo software (Flowjo, Tree Star, Ashland, OR, USA).

### Real-time PCR

Total RNA from heart tissues was extracted with TRIzol Reagent (Invitrogen, Gaithersburg, MD,USA), and then converted into cDNA with M-MuLV reverse transcriptase (Fermentas International Inc., Burlington, ON, Canada) according to the manufacturer’s instructions. Real time-polymerase chain reaction (RT-PCR) was performed using an ABI 7500 Sequence Detection System (Applied Biosystems, Foster City, CA, USA) using SYBR green. To measure the viral loads in heart tissues, the total RNA was reverse transcribed to cDNA using a CVB3-specific positive-strand RNA primer (5’-CACCGGATGGCCAATCCA-3’) or a negative-strand RNA primer (5’-GCGAAGAGTCTATTGAGCTA-3’) and then subjected to SYBR Green real-time PCR using CVB3 primers. The primer sequences used are shown in Table 1. The relative gene expressions were normalized to the level of β-actin transcripts and quantified by the 2^-△△CT^ method. All reactions were performed in at least duplicate for each sample.

**Table 1:** Real-time PCR primers

Gene	Primer sequence (5′-3′)
IL-27RA	Forward: CAAGAAGAGGTCCCGTGCTG
	Reverse: TTGAGCCCAGTCCACCACAT
IL-17A	Forward: CTCCAGAAGGCCCTCAGACTAC
	Reverse: AGCTTTCCCTCCGCATTGACACAG
IL-22,	Forward: CATGCAGGAGGTGGTACCTT
	Reverse: CAGACGCAAGCATTTCTCAG
ROR-γt	Forward: ATGACATGCACCTGGAACACT
	Reverse: TGTGAGTTCTCCATGCCTAGG
CVB3	Forward: ATCAAGTTGCGTGCTGTG
	Reverse: TGCGAAATGAAAGGAGTGT
β-actin	Forward: CACCATTGGCAATGAGCGGTTC
	Reverse: GTAGTTTCGTGGATGCCACAG

### Western blotting

About 20 μg of total protein form heart tissues was extracted and separated by 10 % SDS-PAGE, transferred onto polyvinylidene fluoride membranes, and then reacted with primary antibodies against Anti-IL-27RA (1:500) and β-actin (1:1000) (all from R&D Systems, Minneapolis, MN, USA). After being extensively washed with PBS containing 0.1 % Triton X-100, the membranes were incubated with alkaline phosphatase-conjugated goat anti-rabbit antibody for 30 min at room temperature. The bands were visualized using 1-step TM NBT/BCIP reagents (Thermo Fisher Scientific, Rockford, IL, USA) and detected by an Alpha Imager (Alpha Innotech, San Leandro, CA, USA).

### Cytokine ELISAs

Blood was collected via retro-orbital bleeding and serum was separated. Freshly isolated heart tissue was ground to a fine powder under liquid nitrogen. Each sample (100 mg of powdered tissue) was homogenized in 0.5 mL of RIPA buffer and then centrifuged in a cooled microcentrifuge for 8 min. The supernatants were then subjected to ELISA. The amounts of IL-27, IL-17A, IFN-γ, TNF-α and IL-6 were determined by ELISA kits (R&D Systems, Minneapolis, MN, USA) according to the manufacturer’s instructions. All samples were measured in triplicate.

### Statistical analysis

All Data were presented as means ± SEM. Differences between experimental groups were analyzed using an unpaired Student’s t-test. Correlations were determined by Spearman rank correlation coefficients. Survival was estimated by the Kaplan-Meier method and compared by the log-rank test. All data were analyzed with GraphPad Prism version5.0 (GraphPad Software Inc.). *P* < 0.05 was considered significant difference.

## Additional file

Additional file 1: Figure S1. IL-27 did not affect the body weight loss and survival in mice not-infected with the CVB3. Male BALB/c mice were administered i.p. with PBS at day 0; then mice were injected i.p. with rmIL-27 or PBS on day 0 and 5 after CVB3 infection. The survival rates (A), body weight (B) were monitored. Data are showed as the means ± SEM. Each group contained ten mice. (TIF 819 kb)
